The article "11,670 whole-genome sequences representative of the Han Chinese population from the CONVERGE project" was retracted in 2020. Reason: no approval from a third party.

# 11,670 whole-genome sequences representative of the Han Chinese population from the CONVERGE project

**DOI:** 10.1038/sdata.2017.11

**Published:** 2017-02-14

**Authors:** Na Cai, Tim B. Bigdeli, Warren W. Kretzschmar, Yihan Li, Jieqin Liang, Jingchu Hu, Roseann E. Peterson, Silviu Bacanu, Bradley Todd Webb, Brien Riley, Qibin Li, Jonathan Marchini, Richard Mott, Kenneth S. Kendler, Jonathan Flint

**Affiliations:** 1 Wellcome Trust Centre for Human Genetics, OX3 7BN Oxford, UK; 2 Wellcome Trust Sanger Institute, Wellcome Genome Campus, CB10 1SA Hinxton, Cambridge, UK; 3 European Molecular Biology Laboratory, European Bioinformatics Institute, Wellcome Genome Campus, CB10 1SD Hinxton, Cambridge, UK; 4 Virginia Institute for Psychiatric and Behavioral Genetics, Virginia Commonwealth University, Richmond, Virginia 23298, USA; 5 BGI-Shenzhen, Shenzhen, Guangdong 518083, China; 6 Department of Statistics, University of Oxford, Oxford OX1 3TG, UK; 7 UCL Genetics Institute, University College London, London WC1E 6BT, UK; 8 Center for Neurobehavioral Genetics, Semel Institute for Neuroscience and Human Behavior, University of California, Los Angeles, Los Angeles, California 90095-1761, USA

**Keywords:** Genetic predisposition to disease, Genetic variation, Genetic markers, DNA sequencing

## Abstract

The China, Oxford and Virginia Commonwealth University Experimental Research on Genetic Epidemiology (CONVERGE) project on Major Depressive Disorder (MDD) sequenced 11,670 female Han Chinese at low-coverage (1.7X), providing the first large-scale whole genome sequencing resource representative of the largest ethnic group in the world. Samples are collected from 58 hospitals from 23 provinces around China. We are able to call 22 million high quality single nucleotide polymorphisms (SNP) from the nuclear genome, representing the largest SNP call set from an East Asian population to date. We use these variants for imputation of genotypes across all samples, and this has allowed us to perform a successful genome wide association study (GWAS) on MDD. The utility of these data can be extended to studies of genetic ancestry in the Han Chinese and evolutionary genetics when integrated with data from other populations. Molecular phenotypes, such as copy number variations and structural variations can be detected, quantified and analysed in similar ways.

## Background & Summary

CONVERGE^1^ is the largest whole-genome sequencing cohort representative of the Han Chinese population to date. It is also the most comprehensive collection of sequence variants from any non-Caucasian population.

The 1000 Genomes Project^2–4^, Hapmap project^5^, the Human Genome Diversity Project^6^ (HGDP) and most recently assembly of many population based cohorts in the Haplotype Reference Consortium have enabled the study of genetic diversity in human populations and the building of population reference panels for checking any new cohorts against as well as genotype imputation. Despite these efforts, most genetic studies have mostly been conducted in European and African populations. Examples of relatively large GWAS on East Asian populations on schizophrenia^7^, IgA nephrology^8^, prostate cancer^9^ and systemic lupus erythematosus^10^ have discovery sample sizes below 2,000 cases. In comparison, more diseases are studied using the GWAS method on populations of European descent, more cohorts were collected by independent groups for each disease, many of them are aggregated in large consortiums for joint analysis, and as such have sample sizes at least a scale of magnitude larger. Some examples include the Wellcome Trust Case Control Consortium Phase 1 (ref. 11) (WTCCC-1, all samples of European descent), the DIAGRAM Consortium for type-II diabetes^12^ (34,840 cases and 114,981 controls, mostly of European descent), the CardioGRAM Consortium^13^ for coronary artery disease (60,801 cases and 123,504 controls, mostly of European descent), the CHARGE Consortium^14^ (38,000 samples, all analyses restricted to Europeans or European Americans) and most recently, the UKBiobank and 23andMe datasets each containing hundreds of thousands of samples and numerous quantitative and qualitative traits reflective of human physiology and lifestyle.

Few methods^15^ had been developed to analyze cross population data, and significant success has only recently been achieved in meta-analysis^16^. Such successes have also been limited to genetic loci that have similar allele frequency distributions in different populations. Most resources such as recombination maps, linkage disequilibrium (LD) maps, and particular disease related gene annotations^17–19^ being developed with and drawing information mostly from European populations, and population specific ones are increasing in numbers but still exceptions^20^ rather than the norm. CONVERGE samples^1^ consist of cases of recurrent MD collected from 58 provincial mental health centres and psychiatric departments of general medical hospitals in 45 cities and 23 provinces of China. A similar number of controls are recruited from patients undergoing minor surgical procedures at general hospitals (37%) or from local community centres (63%). While these data are collected for the investigation of genetics of severe recurrent MDD in the Han Chinese population, sequence data from this dataset are a resource for population genetics studies on the Han Chinese population. In particular, these data can be used as a reference panel for future design of genotyping arrays specific to the Han Chinese population, and as comparison with other populations in the investigation of human evolution and migration. LD maps, recombination maps and allele frequency spectrums can be generated from this dataset for use as reference for Han Chinese or other related East Asian populations.

In addition, the presence of mitochondrial sequence data at an average coverage of 102X in all CONVERGE samples^21,22^ can be used to trace the maternal lineage of the Han Chinese population. We have previously reported mitochondrial DNA copy number is under genetic control^22^; there are potentially other molecular traits detectable from whole-genome sequencing data under genetic control.

CONVERGE is the largest genetic resource derived from next generation whole genome sequencing (WGS) and it showcases the utility of low-coverage WGS in providing high quality genotypes for GWAS at common variant sites. We outline the tested practices in sequence data processing, variant calling, variant filtering, imputation and downstream quality control, setting a benchmark for future studies using low coverage WGS for GWAS and other genetic analyses.

## Methods

### Sample collection

CONVERGE collected cases of recurrent MDD from 58 provincial mental health centres and psychiatric departments of general medical hospitals in 45 cities and 23 provinces of China. Controls were recruited from patients undergoing minor surgical procedures at general hospitals (37%) or from local community centres (63%). Cases were excluded if they had a pre-existing history of bipolar disorder, psychosis or mental retardation. Cases were aged between 30 and 60 and had two or more episodes of MDD meeting DSM-IV criteria^23^ with the first episode occurring between 14 and 50 years of age, and had not abused drugs or alcohol before their first depressive episode. All subjects were interviewed using a computerized assessment system. Interviewers were postgraduate medical students, junior psychiatrists or senior nurses who had gone through at least a week of training by the CONVERGE team. The diagnosis of MDD was established with the Composite International Diagnostic Interview (CIDI) (WHO lifetime version 2.1; Chinese version), which utilized DSM-IV criteria. The interview was translated into Mandarin by a team of psychiatrists in Shanghai Mental Health Centre, with the translation reviewed and modified by members of the CONVERGE team.

### DNA sequencing

DNA was extracted from saliva samples using the Oragene protocol. A barcoded library was constructed for each sample. Sequencing reads obtained from Illumina Hiseq machines were aligned to Genome Reference Consortium Human Build 37 patch release 5 (GRCh37.p5) with Stampy (v1.0.17)^24^ using default parameters, after filtering out reads containing adaptor sequencing or consisting of more than 50% poor quality (base quality<=5) bases. Samtools (v0.1.18)^25^ was used to index the alignments in BAM format^25^ and Picardtools (v1.62) was used to mark PCR duplicates for downstream filtering. The Genome Analysis Toolkit’s (GATK, version 2.6)^26^ Base quality score recalibration (BQSR) was then applied to the mapped sequencing reads using BaseRecalibrator in Genome Analysis Toolkit (GATK, basic version 2.6)^26^ with the known insertion and deletion (INDEL) variations in 1000 Genomes Projects Phase 1 and known single nucleotide polymorphisms (SNPs) from dbSNP (v137, excluding all sites added after v129) excluded from the empirical error rate calculation. GATKlite (v2.2.15)^26^ was then used to output sequencing reads with the recalibrated base quality scores while removing reads without the ‘proper pair’ flag bit set by Stampy (1–5% of reads per sample) using the --read_filter ProperPair option (if the ‘proper pair’ flag bit is set for a pair of reads, it means both reads in the mate-pair are correctly oriented, and their separation is within 5 standard deviations from the mean insert size between mate-pairs).

### Calling and imputation of genotypes at SNPs included in GWAS

Variant discovery and genotyping (for both SNPs and INDELs) at all polymorphic SNPs in 1000G Phase1 East Asian (ASN) reference panel^3^ was performed simultaneously using post-BQSR sequencing reads from all samples using the GATK’s UnifiedGenotyper (version 2.7-2-g6bda569) using option --genotype_likelihood_model BOTH and default annotation outputs for variant calls. dbSNP v137 rsids were used to fill in the variant ID column of the result variant call format (VCF) files using the --dbSNP option. Variant quality score recalibration (VQSR) was then performed with GATK’s VariantRecalibrator (v2.7-4-g6f46d11) in SNP variant calls using the SNPs in 1000 Genomes Phase 1 ASN Panel^3^ as the known, truth and training sets with a prior of 15.0, and the following default annotations: -an QD -an HaplotypeScore -an MQRankSum -an ReadPosRankSum -an FS -an MQonly. A sensitivity threshold of 90% to SNPs in the 1000G Phase1 ASN panel was applied for SNP selection for imputation after optimizing for Transition to Transversion (TiTv) ratios in SNPs called. Genotype likelihoods (GLs) were calculated at selected sites using a sample-specific binomial mixture model implemented in SNPtools (version 1.0)^27^, and imputation was performed at those sites without a reference panel using BEAGLE (version 3.3.2)^28^. A second round of imputation was performed with BEAGLE on the same GLs, but only at biallelic SNPs polymorphic in the 1000G Phase 1 ASN panel using the 1000G Phase 1 ASN haplotypes as a reference panel. A final set of allele dosages and genotype probabilities was generated from these two datasets by replacing the results in the former with those in the latter at all sites imputed in the latter. We then applied a conservative set of inclusion threshold for SNPs for genome-wide association study (GWAS): (a) *P*-value for violation HWE > 10^−6^, (b) Information score > 0.9, (c) MAF in CONVERGE > 0.5% to arrive at the final set of 6,242,619 SNPs for individual genotype analsyses.

### Haplotype calling

The genotypes derived from Beagle imputation were phased using Shapeit (version 2, revision 790)^29^. Genetic maps were obtained from the Impute2 (ref. 30) website. Chromosomes 13–22 and X were phased using 12 threads and default parameters. Chromosomes 1–12 were phased using 12 threads in four chunks that overlap by 1MB. The phased chunks were ligated together using ligateHAPLOTYPES, available from the Shapeit website.

### Ethical approval

The study protocol was approved centrally by the Ethical Review Board of Oxford University (Oxford Tropical Research Ethics Committee) and the ethics committees of all participating hospitals in China. All interviewers were mental health professionals who are well able to judge decisional capacity. The study posed minimal risk (an interview and saliva sample). All participants provided their written informed consent.

## Data Records

### Sequence data

Sequencing data of 11,670 samples in paired FASTQ files are available from the European Nucleotide Archive (ENA) at Study and Short Read Archive Accession PRJNA289433 (Data Citation 1). Data totals about 100 terabytes (TB); after download, alignment of raw sequence data in paired FASTQ format to Genome Reference Consortium Human Build 37 patch release 5 (GRCh37.p5) with BWA takes not more than 2 h per FASTQ file (4 h per pair) and less than 5 gigabytes (GB) of RAM per process. Once in BAM format, preprocessing steps can be parallelized per sample using less than 12GB of RAM and 2 h on a single processor.

### SNP variant calls from sequence data

A list of high quality SNP variant sites^1^ with major and minor alleles and allele frequencies in both the CONVERGE cohort and 1000 Genomes Phase 1 ASN samples in variant call format (VCF) is provided through Figshare (Data Citation 2).

### Imputation and genotypes

We imputed genotype probabilities and obtained alternative allele dosages at 22,847,544 SNPs from all autosomes and chromosome X including 20,539,441 SNPs in the CONVERGE cohort and all polymorphic sites in the 1000 Genomes ASN Panel on all 11,670 CONVERGE samples, as detailed in Cai *et al.*^1^ (Data Citation 2). After applying stringent quality controls, we obtained 10,640 samples (5,303 cases of MDD, 5,337 controls) for inclusion in GWAS of MDD^1^. We have submitted all imputed genotypes at 20,539,441 SNPs of these 10,640 samples passing quality control in VCF format to the European Variations Archive (EVA), Accession PRJNA289433 (same Accession as the sequence data, see ‘Analysis Files’ on ENA study page, Data Citation 3); access will be brokered through the EVA with standard application procedures. SNPs with imputation information score below 0.95 (a higher threshold than we had used for our GWAS analysis) are marked ‘INFO0.95’ instead of ‘PASS’. Minor allele frequency, *P* value for violation of Hardy-Weinberg equilibrium and imputation information score are also present in the INFO column of the VCFs. As CONVERGE is part of Phase 2 of the Haplotype Reference Consortium^31^ (HRC), these data will also be available in the near future through the HRC.

### Genome wide association study summary statistics

GWAS on MDD and mitochondrial DNA copy number quantified from sequencing data are published^1,22^; summary statistics for GWAS on MDD is available from the Psychiatric Genomics Consortium (https://www.med.unc.edu/pgc/files/resultfiles/converge.MDD.summary_stats.2Sep2015.tbl.gz) and on Figshare (Data Citation 4) and that of mitochondrial DNA copy number for all common SNPs (>5% MAF) is available on Figshare (Data Citation 5). All phenotypes are currently under analysis, interested research groups and individuals are welcome to contact us directly for collaborations and access.

## Technical Validation

These methods are expanded versions of descriptions in our related work Cai *et al.*^1^.

### Whole genome NGS on 11,670 samples

The coverage of sequencing is the number of times, on average, a single site in the genome is covered by sequencing reads. For each sample in CONVERGE, the average sequencing coverage over the nuclear genome is 1.7x, and that on the mitochondrial genome is 102x (Fig. 1).

### Variant calling and variant quality recalibration

Sets or ‘tranches’ of SNPs with increasing VQSLOD scores (increasing stringency in exclusion of outliers and concomitant decreasing sensitivity to known SNPs) from VQSR (Methods) were generated at the specified sensitivities to known SNPs using the –tranche option: -tranche 100.0 -tranche 99.9 -tranche 99.0 -tranche 98.0 -tranche 95.0 -tranche 90.0 -tranche 89.0 -tranche 87.0 -tranche 85.0 -tranche 80.0 -tranche 79.0. Transition-to-transversion (TiTv) ratios were calculated for each tranche. Table 1 summarizes this information. A sensitivity to known SNPs of 90.0% was chosen for the inclusion of novel SNPs in downstream analyses, as it balances optimization of TiTv ratio in novel SNPs with retaining as many potential novel SNPs as possible so as not to lose variant information.

This gave a total of 21,356,798 (9,053,391 known in 1000 Genomes Phase 1 ASN Panel and 11,486,024 novel), biallelic SNPs identified from all chromosomes and unassembled contigs. 20,539,441 SNPs from the autosomes and chromosome X were put forth for imputation of genotype probabilities and downstream analyses. All known sites in 1000 Genomes Phase 1 ASN panel were included in all further analyses regardless of whether they were identified as polymorphic in CONVERGE, and their VQSLOD scores if they were identified as polymorphic in CONVERGE. Numbers of SNPs imputed in each chromosome and the percentage of SNPs in each category are shown in Table 2.

### Imputation quality

#### Using high coverage (10x) sequencing

Nine samples in CONVERGE were sequenced to an average of 10x coverage using the same Illumina Hiseq platform used for the low-coverage sequencing samples. Mapping and processing of the 10x sequencing reads were performed in an identical fashion as the low-coverage sequences. Variant calling (for both SNPs and INDELs) was performed on the high coverage dataset using sequencing reads from all nine samples with UnifiedGenotyper in GATK (v2.7-2-g6bda569) using option --genotype_likelihood_model BOTH and default annotation outputs for variant calls. dbSNP v137 rsids are used to fill in the variant ID column of the result variant call format (VCF) files using the --dbSNP option.

Variant quality score recalibration (VQSR) was performed using two different training sets. The first VQSR was performed using SNP variant calls using the SNPs in 1000 Genomes Phase 1 ASN Panel as the known, truth and training sets with a prior of 15.0 and the default annotations just like it was done for the raw variant calls from the low coverage data, but with two maximum Gaussians for building the positive model instead of one, with the --maxGaussian option. The second VQSR was performed using SNPs from the HumanOmniZhongHua-8 (v1.0) BeadChip. Sets or ‘tranches’ of SNPs with increasing VQSLOD scores (increasing stringency in exclusion of outliers and concomitant decreasing sensitivity to known SNPs) were generated at the specified sensitivities to known SNPs using the –tranche option: -tranche 100.0 -tranche 99.9 -tranche 99.0 -tranche 98.0 -tranche 95.0 -tranche 90.0 -tranche 89.0 -tranche 87.0 -tranche 85.0 -tranche 80.0 -tranche 79.0. Transition to Transversion (TiTv) Ratio was calculated for each tranche. A sensitivity to known SNPs in the Zhonghua chip of 90.0% was chosen for the inclusion of novel SNPs in downstream analyses as it balances optimization of TiTv ratio in novel SNPs while retaining as many potential novel SNPs as possible to not lose variant information. This gave a total of 5,914,716 (5,272,185 known in 1000 Genomes Phase 1 ASN Panel and 642,525 novel) biallelic SNPs identified in high coverage sequencing data with which we are able to check for squared Pearson correlation coefficient (r^2^) and concordance with imputed allele dosages and hard-called genotypes of the same samples respectively.

We calculated the percentage concordance between hard-called genotypes from imputed genotype probabilities (where the genotype with the maximum imputed genotype probability>0.9 was called) and genotypes called from the 10x coverage sequencing data at all imputed variant sites for each of the nine samples. The mean concordance per sample across all sites was 98.1% (s.e.=0.12%) and the percentage concordance calculated for each alternative allele frequencies was shown in Fig. 2.

We also calculated r^2^ between imputed allele dosages and genotypes from the 10x coverage sequencing data at all imputed variant sites for each of the nine samples. The mean r^2^ per sample across all sites was 0.938 (s.e.=0.003). The r^2^ calculated for each alternative allele frequencies is shown in Fig. 3.

Supplementary Table 1 from Cai *et al.*^1^ combines all these information and shows the mean percentage concordance and Pearson r^2^ among 9 samples for each genotype class (homozygous reference, heterozygous and homozygous alternative) for each alternative allele frequency bin.

#### Using HumanOmniZhongHua-8 (v1.0) BeadChip on 72 samples

72 samples from CONVERGE were genotyped on the Illumina HumanOmniZhongHua-8 (v1.0B) BeadChip which contains 898,122 SNPs, optimized for the Chinese population using tag SNPs from all three HapMap phases and the 1000 Genomes Project. Sample genotypes with GenCall score of 0.15 or lower were considered no-calls.

857,766 out of the 895,623 SNPs on the array were included in our imputation (95.77%). Upon examining, why 37,857 SNPs on the array were not imputed, we found that SNPs that were on the array, but not imputed, were not polymorphic in either CONVERGE samples or 1000 Genomes Phase 1 ASN panel. None of the 72 samples genotyped were polymorphic at these 37,857 sites. Table 3 shows the number of SNPs genotyped on the Zhonghua array on each chromosome, and the call rate among the 72 samples on each chromosome. 855,132 SNPs that showed biallelic polymorphism in CONVERGE or the 1000 Genomes Phase1 ASN Panel and passed genotyping quality filters were used for comparison with imputation results. We calculated the percentage concordance (Fig. 4) and Pearson r^2^ (Fig. 5) between hard-called genotypes and allele dosages from imputation with genotype calls from the ZhongHua8 genotyping array for all 855,132 SNPs on 72 samples. The overall percentage concordance for all 855,132 imputed SNPs genotyped on the array was 98.0% (s.e.=0.04%) and the overall r^2^ was 0.974 (s.e.=0.0005).

Supplementary Table 2 from Cai *et al.*^1^ shows the mean percentage concordance and Pearson R^2^ among 72 samples for each genotype class (homozygous reference, heterozygous and homozygous alternative) for each alternative allele frequency bin. At all alternative allele frequency bins between 1 to 99%, the mean percentage concordances were above 96% and the mean R^2^s were above 0.87.

#### Using Sequenom at 21 sites

11,669 samples out of all CONVERGE samples were genotyped at 21 random sites in the genome using a custom Sequenom SpectroCHIP (1 sample was not genotyped as there was not enough DNA of adequate quality for genotyping on the Sequenom platform). Mass spectra were collected using the MassARRAY system mass spectrometer and TYPER4.0 was used to assess the reliability of genotype calls generated by SpectroREAD from the mass spectra. Default genotype call inclusion criteria were used.

Just as we had compared imputed results with genotypes called directly from 10x coverage sequencing and the Illumina HumanOmniZhongHua Beadchip, we calculated the percentage concordance and r^2^ between hard-called genotypes and allele dosages from imputation with genotype calls from the Sequenom for each of the 21 sites that were genotyped. An r^2^ of 0.988 and concordance of 98.19% were obtained for the 21 sites. Per site r^2^ (mean=0.985) and percentage concordance (mean=98.16%) are shown Table 4 (also Supplementary Table 3 of Cai *et al.*^1^) along with the alleles and MAF of each site.

### Selection of samples for genetic analyses

#### Sample contamination

We performed a range of quality control filters on all 11,670 samples and selected only those samples with high-quality sequencing results and imputed genotype probabilities for downstream analysis.

We first looked into both the nuclear genome and mitochondrial genome for an excess of variants called, since this would indicate cross-sample contamination due to technical issues during sequencing. We quantified the number of singleton variants called in the genic regions of the nuclear genome (Methods) and found a mean of 71.55 singletons variants in exon regions across the whole genome supported by more than 2 sequencing reads passing sequencing quality controls per sample. While most samples fall in a normal distribution with mean of 71.55 singletons, others had excess singletons, which could be indicative of poor DNA quality that compromised sequencing and mapping qualities. We excluded 117 samples with a number of singletons greater than the 99th percentile (237.62 singletons).

We then asked if there were any samples with an excess of heteroplasmic mutations in the mitochondrial DNA per sample. As the DNA for all individuals recruited in CONVERGE were extracted from saliva samples, which would also contain the oral microbiome, external DNA contamination levels could be told from number of mismatches in mapped reads at regions of the genomes where the human genome was similar to bacterial genomes. The mitochondrial DNA in human genome, a 16 kb circular DNA, is one of such instances. Mitochondrial DNA is inherited only from the mother and there is a strict bottleneck in the female germline for mitochondrial DNA, usually only one clonal copy of mitochondrial DNA is inherited at a time. Heteroplasmic variations in the mitochondrial genome (where two or more alleles are present at a single position in the mitochondrial genome of a single individual) are rare and usually occurring at low levels. Mismatches that occur in some sequencing reads mapping to the mitochondrial DNA region of the human genome reference in one sample would therefore indicate either a rare event heteroplasmy, or a contamination from similar DNA sequences of bacterial origins. Samples with excessive numbers of heteroplasmic sites can therefore be suspected as having a higher than normal level of bacterial contamination, and the conservative approach would be to filter them out to ensure the quality of sequencing, and all downstream analyses.

Coverage of the mitochondrial genome is on average 102X, making it possible to obtain high quality sequence for this part of the genome. We called a mean of 15.70 heteroplasmic sites per sample, and 116 samples were found to have greater than the 99th percentile of number of heteroplasmic sites. Of these 116 samples, 26 were already discarded for having excess nuclear genome singletons; we excluded the additional 90 from further analysis.

#### Sample relatedness

Varying levels of relatedness could cause inflated *P*-values and even false positive results in GWAS, as alleles inherited together due to high relatedness but not related to etiology of disease could appear so in association testing. To exclude duplicates and first degree relatives from our sample for GWAS, we calculated the proportion IBD (PIHAT, estimated as P(IBD=2)+0.5*P(IBD=1)) for every pair of samples in CONVERGE using LD pruned SNPs (LD<0.5). We excluded all pairs of samples (392 samples in total) whose PIHAT exceeded 0.5 and P(IBD=1) exceeded 0.75 from further analyses.

Finally, we also excluded 29 samples with fewer than 90% of imputed sites with maximum genotype probabilities>0.9, and 402 samples with incomplete phenotype information. We used the remaining set of 10,640 samples (5,303 cases of MDD, 5,337 controls) for GWAS on MDD and mitochondrial DNA levels (Data Citation 4 and Data Citation 5).

## Usage Notes

CONVERGE is the largest well-curated, high quality low-coverage WGS dataset from a single study and a single population where all samples are from the same ethnic group. Although sequencing was performed at low coverage, we have shown good quality genotypes can be obtained through recalibration of sequencing base qualities, filtering of variants based on sensitivity to known variants, imputation using a two-step approach, and finally strict quality control over imputed genotypes. We have also shown robust ways of identifying and removing potentially contaminated samples using sequencing data, particularly where the source of DNA was saliva. We have ensured there are no related individuals in this dataset for downstream genetic analysis, and we recommend using genotypes of SNPs with high imputation information scores, available in the VCF we provide through EVA (Data Citation 3) in future analyses. We encourage all users of CONVERGE data to use and expand upon on these quality control measures especially when performing analyses on rare, copy number and structural variants, for which we do not currently have gold standards in low coverage WGS. Development of methods and best practices for these purposes can enable more economical sequencing of large cohorts, and the usage of existing data to the fullest.

The CONVERGE project has the aim of studying MDD in a homogenous population where genetic ancestry and cultural diversity minimally confound genetic effects. Hospital staff, trained to use computer-assisted interviews, obtained highly detailed information on clinical symptoms, comorbidities, personality traits, social support, socio-economic status, life style, and major stressful life events. All cases of MDD collected in CONVERGE had severe and recurrent MDD not concurrent with other major illnesses (85% of cases of MDD in CONVERGE come under the severe subtype with somatic symptoms, Melancholia). The use of screened controls limited the possibility of including undiagnosed cases of MDD in the study. These, together with strict inclusion criteria for ancestry, age (between 30 to 60) and sex (only females) of all samples in CONVERGE, made CONVERGE the most homogenous and extensively phenotyped cohort of severe, recurrent MDD and matched controls to date.

MDD is a highly heterogeneous disease with different ages of onset and physiological symptoms, prevalence between sexes, definitions across cultural contexts and diagnostic instruments. In addition to heterogeneity in the disease presentation, misdiagnoses and biases in self-reporting further contribute to heterogeneity in studies with less detailed enquiry, documentation and classification of MDD phenotypes. Until recently, GWAS has not been able to uncover genetic loci associated with MDD due to the complex genetic architecture^32^ (commonly thought to consist of small effects from numerous common genetic variants) compounded with heterogeneity in disease identification and characteristics. The estimated number of samples needed for uncovering a genetic locus associated with this heterogenous disease was 50,000 cases and a similar number of controls. In CONVERGE we have shown that using stringent criteria and deep phenotyping to minimise misdiagnosis and biases in self-reporting, we were able to find and replicate two genetic associations to MDD using a tenth of the estimated sample size. Thus, in some cases, dissection of disease etiology through studying clearly defined and rigorously collected phenotypes can lead to a substantial increase in power to detect genetic effects. We note the contrast in strategy with a recent study using data from 23andMe that reported 15 genetic associations with 30 times our sample size and a yet bigger departure from our definition of MDD^33^. It will take further investigations to know if and how these new genetic associations from a large but heterogenous cohort may contribute to genetic heterogeneity in MDD.

## Additional information

**How to cite this article**: Cai, N *et al.* 11,670 whole-genome sequences representative of the Han Chinese population from the CONVERGE project. *Sci. Data* 4:170011 doi: 10.1038/sdata.2017.11 (2017).

**Publisher**’**s note**: Springer Nature remains neutral with regard to jurisdictional claims in published maps and institutional affiliations.

## Supplementary Material



## Figures and Tables

**Figure 1:** Sequencing coverage per sample in CONVERGE. This figure shows the mean sequencing coverage per site in the nuclear and mitochondrial genome per sample for 11,670 samples in CONVERGE; the mean sequencing coverage over the nuclear genome is 1.7X and that over the mitochondrial genome is 102X.

**Figure 2:** Percentage concordance between hard-called genotypes from imputed genotype probabilities and genotypes called from 10x coverage sequencing in nine samples. This figure shows the percentage concordance between genotypes from imputation (hard-called as the genotype with the maximum imputed genotype probability, barring those where the maximum genotypes probability was smaller than 0.9 in which case the genotypes was considered missing) and genotypes directly called from 10x coverage sequencing data in nine samples. Each box contains data points for nine samples; the vertical axis shows the percentage of SNPs per sample in each alternative allele frequency bracket (horizontal axis) with concordant genotypes between the two datasets.

**Figure 3:** Aggregate Pearson r^2^ between imputed allele dosages and genotypes called from 10x coverage sequencing in nine samples. This figure shows the aggregate Pearson r^2^ between imputed alternative allele dosages with genotypes called directly from 10x coverage sequencing data in nine samples. Each box contains data points for nine samples; the vertical axis shows aggregate Pearson r^2^ of all SNPs in each alternative allele frequency bracket (horizontal axis) with concordant genotypes between that imputed alternative allele dosages and directly called from 10x coverage sequencing data.

**Figure 4:** Percentage concordance between hard-called genotypes from imputed genotype probabilities and genotypes from the Illumina HumanOmniZhongHua Beadchip in 72 samples. This figure shows the percentage concordance between genotypes from imputation (hard-called as the genotype with the maximum imputed genotype probability, barring those where the maximum genotypes probability was smaller than 0.9 in which case the genotypes was considered missing) and genotypes directly called from Illumina HumanOmniZhongHua Beadchip in 72 samples. Each box contains data points for nine samples; the vertical axis shows the percentage of SNPs per sample in each alternative allele frequency bracket (horizontal axis) with concordant genotypes between the two datasets.

**Figure 5:** Aggregate Pearson r^2^ between imputed allele dosages and genotypes called from Illumina HumanOmniZhongHua Beadchip in 72 samples. This figure shows the aggregate Pearson r^2^ between imputed alternative allele dosages with genotypes called directly from 10x coverage sequencing data in nine samples. Each box contains data points for nine samples; the vertical axis shows aggregate Pearson r^2^ of all SNPs in each alternative allele frequency bracket (horizontal axis) with concordant genotypes between that imputed alternative allele dosages and directly called from Illumina HumanOmniZhongHua Beadchip in 72 samples.

**Table 1:** Transition-Transversion (TiTv) ratio for known and novel SNPs discovered in CONVERGE in different tranches of sensitivities to known SNPs in 1000 Genomes Phase 1 ASN Panel.

**Sensitivity to Known SNPs (%)**	**Number of SNPs**		**TiTv Ratio**	
	**Known**	**Novel**	**Known**	**Novel**
79	7946865	9361731	2.1783	2.1998
80	8047459	9502607	2.1786	2.2011
85	8550425	10357018	2.1817	2.204
87	8751611	10853838	2.1838	2.2042
89	8952798	11310561	2.1862	2.1961
90	9053391	11486024	2.187	2.1868
95	9556357	13089943	2.1849	1.9637
98	9858137	15716679	2.1759	1.6553
99	9958730	17362038	2.1721	1.5296
99.9	10049264	20940831	2.1683	1.353
100	10059324	22722016	2.168	1.2839
This table shows the results of VQSR on all SNPs called in CONVERGE using default annotations in GATK and biallelic SNPs in 1000 Genomes Phase 1 ASN Panel as ‘known’, ‘true’, and ‘training’ sets. The first column shows the tranche defined by sensitivity to known set, the second and third column shows the number of known and novel SNPs in CONVERGE falling into each tranche, and the last two columns show the TiTv ratio of known and novel SNPs in each tranche respectively.				

**Table 2:** Imputed SNPs in CONVERGE.

**Chr**	**All Imputed**	**Known in 1000 Genomes Phase 1 ASN Panel**			**Novel in CONVERGE**					**Used in GWAS**	
		**Imputed**	**CONVERGE**		**Not in CONVERGE**		**% of Imputed**	**Count**	**% of Imputed**	**Count**	**% of Imputed**
			**Count**	**(%)**	**Count**	**(%)**					
chr1	1906566	1049943	709178	67.54	340765	32.456	55.07	856623	44.93	473126	24.82
chr2	2080626	1141277	768281	67.32	372996	32.682	54.85	939349	45.15	504269	24.24
chr3	1730976	971680	660330	67.96	311350	32.042	56.14	759296	43.87	444601	25.69
chr4	1683635	963695	655100	67.98	308595	32.022	57.24	719940	42.76	452165	26.86
chr5	1552865	866733	586899	67.71	279834	32.286	55.82	686132	44.19	395356	25.46
chr6	1542585	895135	602872	67.35	292263	32.65	58.03	647450	41.97	416919	27.03
chr7	1386630	780333	519815	66.62	260518	33.385	56.28	606297	43.72	357113	25.75
chr8	1352488	743135	500602	67.36	242533	32.636	54.95	609353	45.05	330591	24.44
chr9	1049711	587643	394219	67.09	193424	32.915	55.98	462068	44.02	264762	25.22
chr10	1204931	669919	456560	68.15	213359	31.848	55.6	535012	44.4	310998	25.81
chr11	1203686	662829	443108	66.85	219721	33.149	55.07	540857	44.93	297679	24.73
chr12	1141658	644071	435882	67.68	208189	32.324	56.42	497587	43.59	294448	25.79
chr13	858815	486316	334096	68.7	152220	31.301	56.63	372499	43.37	225668	26.28
chr14	793487	445316	303662	68.19	141654	31.81	56.12	348171	43.88	201734	25.42
chr15	722748	397917	266748	67.04	131169	32.964	55.06	324831	44.94	175810	24.33
chr16	793223	418892	276272	65.95	142620	34.047	52.81	374331	47.19	178608	22.52
chr17	674848	363982	238795	65.61	125187	34.394	53.94	310866	46.07	150405	22.29
chr18	683315	386244	265213	68.67	121031	31.335	56.53	297071	43.48	173158	25.34
chr19	542027	299517	192281	64.2	107236	35.803	55.26	242510	44.74	128700	23.74
chr20	552234	294881	200864	68.12	94017	31.883	53.4	257353	46.6	127726	23.13
chr21	324063	182937	123793	67.67	59144	32.33	56.45	141126	43.55	83062	25.63
chr22	334001	180274	119161	66.1	61113	33.9	53.98	153727	46.03	79845	23.91
chrX	943020	404837	265078	65.48	139759	34.522	42.93	538183	57.07	175876	18.65
Total	25058138	13837506	9318809	67.35	4518697	32.655	55.22	11220632	44.78	6242619	24.91
This table shows the number of imputed SNPs in CONVERGE in each chromosome. The first two columns show the chromosome and total number of SNPs imputed in that chromosome. The next six columns show the composition of these SNPs in relation to the 1000 Genomes Phase 1 ASN Panel: the number of SNPs imputed that were found to be polymorphic in 1000 Genomes Phase 1 ASN Panel, the number and percentage of SNPs polymorphic in CONVERGE, the number and percentage of SNPs not polymorphic in CONVERGE, and the percentage of SNPs in 1000 Genomes Phase 1 ASN Panel among all imputed SNPs. The following two columns show the number and percentage of imputed SNPs that were novel in CONVERGE. The final two columns show the number and percentage of imputed SNPs that were included in the GWAS for MDD.											

**Table 3:** **SNPs genotyped per chromosome on Illumina HumanOmniZhongHua Beadchip.**

**Chromosome**	**All Array SNPs**	**No Calls**	**Not Polymorphic**	**Used For Comparison**
chr1	69485	5	3199	66126
chr2	70071	3	2958	66928
chr3	60192	7	2608	57516
chr4	53419	1	2478	50807
chr5	52477	1	2142	50307
chr6	62652	15	2555	59930
chr7	47158	4	1909	45157
chr8	45906	0	1824	44062
chr9	40597	0	1521	38996
chr10	46134	1	1971	44131
chr11	42894	1	1971	40888
chr12	42849	3	1822	40950
chr13	32399	1	1451	30931
chr14	28777	1	1167	27594
chr15	27769	3	1099	26647
chr16	29448	3	1276	28146
chr17	25411	1	1145	24252
chr18	27117	1	1104	26003
chr19	18919	4	956	17942
chr20	21918	2	843	21057
chr21	12613	1	500	12103
chr22	14056	1	480	13538
chrX	23362	1	869	21121
chrY	2041	1208	833	0
chrM	151	0	151	0
chrXY	307	307	0	0
Total	898122	1575	38832	855132
This table shows in the first two columns the chromosome and the number of SNPs on each chromosome on the Illumina HumanOmniZhongHua Beadchip. In the next three columns are the numbers of SNPs with no calls in any of the 72 samples, that are not polymorphic in the 72 samples, and that were polymorphic and genotypes at which were used for comparison with genotypes hard-called from imputed genotype probabilities and imputed alternative allele dosages.				

**Table 4:** **Validation of imputation results with genotypes at 21 sites on custom Sequenom SpectroCHIP on all samples.**

**SNP**	**RSID**	**REF**	**ALT**	**FREQ**	**N Samples**	**Con (%)**	**Pearson r**^**2**^
chr1:11205058	rs1057079	C	T	0.8	11645	99.85	0.998
chr1:47398743	rs3890011	G	C	0.525	11625	99.95	0.999
chr2:141751592	rs13007735	G	A	0.595	11652	99.8	0.998
chr2:204824283	rs10172036	T	G	0.434	9561	94.69	0.957
chr2:99779131	rs2516835	T	C	0.651	11533	99.58	0.997
chr3:186443018	rs1656922	T	C	0.356	11634	99.64	0.996
chr7:47968927	rs2686817	C	A	0.522	11621	99.09	0.992
chr8:143310815	rs11167136	G	A	0.498	11618	98.61	0.987
chr9:125424507	rs70156	A	C	0.5	11632	94.8	0.962
chr10:120917445	rs2275111	G	A	0.707	11651	99.54	0.995
chr10:95279506	rs2293277	A	T	0.565	11506	95.62	0.966
chr12:120995332	rs2292681	G	A	0.767	11653	99.88	0.998
chr13:31233063	rs3742302	G	A	0.153	11651	99.91	0.998
chr14:20665840	rs4981088	G	A	0.507	11508	93.92	0.954
chr15:77344793	rs11737	T	A	0.415	11628	99.69	0.997
chr15:90226947	rs7169981	C	A	0.317	11615	98.92	0.99
chr16:20986506	rs3115438	C	T	0.481	11423	99.79	0.998
chr17:5991344	rs2302836	C	T	0.829	11652	96.52	0.955
chr18:61170721	rs1455556	T	C	0.546	11631	97.73	0.983
chr20:50238545	rs2235862	A	G	0.237	11649	99.8	0.997
chr20:52786219	rs2296241	G	A	0.417	11638	93.99	0.96
The table shows concordance between SNP genotypes from low coverage sequence data and from 21 sites genotyped on a Sequenom SpectroCHIP on all samples. The first five columns show the chromosome and position (SNP), reference allele (REF) on Human Genome Reference GRCh37.p5 and alternative allele (ALT) called in CONVERGE, and the alternative allele frequency (FREQ) in CONVERGE. The next column shows the number of samples (N Samples) with genotypes from Sequenom at each of the 21 sites. The next two columns show the comparison between imputed allele dosages and genotypes from Sequenom at the 21 sites: percentage concordance (Con (%)) was calculated per site between hard-called genotypes from imputed genotype probabilities (where the genotype with the maximum imputed genotype probability > 0.9 was called) and genotypes called from the same samples at the same loci from Sequenom. Pearson r^2^ was also computed per site between imputed allele dosages.							
